This article has been retracted.

# Stimulator of Interferon Genes in Classical Dendritic Cells Controls Mucosal Th17 Responses to Cyclic Dinucleotides for Host Defenses Against Microbial Infections in Gut

**DOI:** 10.3389/fimmu.2018.01085

**Published:** 2018-05-16

**Authors:** Song Liu, Qiuyuan Xia, Xiuwen Wu, Feng Sun, Qiongyuan Hu, Jie Wu, Meng Wang, Qiu Rao, Wenxian Guan

**Affiliations:** ^1^Department of General Surgery, Nanjing Drum Tower Hospital, Nanjing, China; ^2^School of Medicine, Nanjing University, Nanjing, China; ^3^Department of Pathology, Jinling Hospital, Nanjing, China; ^4^Department of General Surgery, Jinling Hospital, Nanjing, China

**Keywords:** stimulator of interferon genes, dendritic cell, Th17, *Salmonella*, cyclic dinucleotides, Crohn’s disease

## Abstract

Cyclic dinucleotides are bacterial signal transducers that bind to host intracellular protein, stimulator of interferon genes (STING) encoded by *Tmem173*. In this study, we demonstrate that STING triggers adaptive immune responses that control Th17 differentiation. Cyclic dinucleotides recognition enables classical dendritic cells (cDCs) that predominantly express CD103 to induce Th17 lymphocytes in an IL-6/IL-1β-dependent manner in gut. STING expression in human lamina propria is associated with the severity of mucosal inflammation and clinical disease activity in patients with Crohn’s disease. Mice deficient in *Tmem173* fail to mount Th17 responses to cyclic dinucleotides or prevent immune evasion of enteroinvasive pathogens. In summary, STING in mucosal cDCs controls Th17 subspecification that is essential for host defenses against microbial infection in gut-associated immune system.

## Introduction

The interaction between intestinal microbiome and host immunity plays a critical role in various autoimmune diseases, including Crohn’s disease (1, 2). Microbial nucleic acid belongs to pathogen-associated molecular patterns that can be recognized by specific sensors in dendritic cells to activate adaptive immunity (3, 4). However, the mechanism that links innate immunity triggered by microbial nucleic acid and functional properties of T cell population in gut-associated mucosal system remains to be elucidated.

Cyclic diguanylate monophosphate (c-di-GMP) is a newly identified second messenger in multiple species of bacteria that is released into cytosol of host cells during microbial infection (5). c-di-GMP is recognized by stimulator of interferon genes (STING) that leads to IRF3 or NF-κB activation (6–8). Mucosal dendritic cells are heterogeneous in origin and function (9, 10) and can induce Th17 cells as well as inducible regulatory T cells as parts of adaptive immune responses to intestinal microbiota (11, 12). However, the underlying signaling mechanism by which this is achieved remains elusive (13). The clinical significance of bacterial cyclic dinucleotides recognition by STING in host antimicrobial defenses awaits full elucidations.

In this study, we show that mucosal classical dendritic cells (cDCs) defined by the transcription factor *Zbtb46* predominantly express CD103. Mucosal cDCs induce Th17 generation through a STING-dependent recognition of foreign cyclic dinucleotides. STING in lamina propria participates in mucosal inflammation and systemic disease activity in human Crohn’s disease. STING-triggered mucosal Th17 responses can prevent immune evasion of enteroinvasive pathogens and are therefore crucial for host antimicrobial defenses in gut.

## Materials and Methods

### Ethics

This study was carried out in accordance with the recommendations of Guidelines for Clinical Trials by the Ethics Committee of Nanjing Drum Tower Hospital. The protocol was approved by the Ethics Committee of Nanjing Drum Tower Hospital. All subjects gave written informed consent in accordance with the Declaration of Helsinki. This study was carried out in accordance with the recommendations of Guidelines for Animal Experiment by the Ethics Committee of Nanjing Drum Tower Hospital. The protocol was approved by the Ethics Committee of Nanjing Drum Tower Hospital.

### Human Samples

Intestine samples from eight adult patients diagnosed as Crohn’s disease were collected from grossly identifiable lesions as well as grossly uninvolved segments during definitive bowel resections. Intestine samples from four adult patients during ileostomy closure served as controls. A written content was obtained from each participant before surgery.

Pathological slides were prepared by fixing specimens in formaldehyde and cutting into 5-µm sections and staining with hematoxylin and eosin. For immunohistochemistry, slides were treated with anti-STING antibody (D2P2F; 13647; Cell Signaling) according to the manufacture’s recommendations. Pixel intensities associated with anti-STING staining were converted to optical densities using Image J software (US National Institutes of Health). An expert gastrointestinal pathologist that was blinded to patient identity reviewed all slides and calculated the pathological score of each participant. The pathological scoring system ranged from 0 (normal) to 15 (most severe of inflammation) including six parameters: cellular infiltration (0–3), loss of goblet cells (0–3), crypt abscess (0–3), epithelial erosion (0–1), hyperemia (0–2), and thickness of mucosa (0–3) (14).

For immunoblotting, the preparation of tissue and protocol were in accordance to published routine method (15). Antibodies for immunoblotting included IRF-3 (D83B9; 4302; Cell Signaling), p-IRF3 (D6O1M; 29047; Cell Signaling), and β-actin (8H10D10; 3700; Cell Signaling). For patients with Crohn’s disease, their preoperative Crohn’s disease activity index (CDAI) score was calculated according to previous literature (16).

### Mice

C57BL/6, *Il17a*^GFP^, *Zbtb46*^GFP^, *Zbtb46*^DTR^, and OT-II mice were purchased from The Jackson Laboratory (Bar Harbor, ME, USA). *Tmem173^−/−^* (*Sting^−/−^*) mice on C57BL/6 background were generated using CRISPR/Cas9 technique in Nanjing Biomedical Research Institute of Nanjing University. All mice were maintained in *H. hepaticus*- and *Pasteurella*-free or specific pathogen-free environment at MARC (Model Animal Research Center of Nanjing University). All animal experiments in this study were undertaken when mice were 6–10 weeks old with protocols approved by the Institutional Subcommittee on Research Animal Care at Nanjing University.

### Bone Marrow Chimeras and Diphtheria Toxin (DT) Depletion

Recipient C57BL/6 mice received whole body irradiation (970cGy). A total of 1 × 10^7^ bone marrow cells from *Zbtb46*^DTR^ or *Zbtb46*^GFP^ mice were injected into recipient mice *via* tail vein. The mice were housed for 8 weeks before subsequent experiments. For DT depletion, 40 ng DT (Sigma-Aldrich, St. Louis, MO, USA) per gram of body weight was injected (i.p.) twice on days 1 and 3 before experiment to specifically deplete the classical DC subsets.

### *In Vivo* Stimulation Assay

To activate STING signaling pathway *in vivo*, 200 nmol/mouse c-di-GMP (VacciGrade) (Invivogen, San Diego, CA, USA) was either injected (i.v.) 18 h before experiment or injected (i.p.) at days 1, 3, and 5 before experiment.

### DC and T Cell Isolation From Spleen, Mesenteric Lymph Nodes (MLN), and Lamina Propria

To isolate DCs from spleen and MLN, the spleen or MLN was incubated with 1 mg/ml collagenase A (Roche Applied Science, Germany) in Dulbecco’s Modified Eagle’s Medium (DMEM; Gibco Life Technology, Gaithersburg, MD, USA) containing 5% fetal bovine serum (Atlanta Biologicals, Flowery Branch, GA, USA) at 37°C in 200 rpm shaker for 30 min. After addition of 5 mM EDTA (Boston Bioproducts, Boston, MA, USA), all cells were passed through a 70 µm nylon cell strainer (Fisher Scientific). A final OptiPrep density centrifugation at ρ = 1.055 g/ml(Axis Shield, Oslo, Norway) yielded DCs.

To harvest cells from small intestine lamina propria (SILP), the small intestine was cut into four pieces and inverted onto polyethylene tubes (Becton Dickinson, Franklin Lakes, NJ, USA). After washing three times with calcium- and magnesium-free PBS (Lonza, Walkersville, MD, USA), the mucus and epithelium were removed by 1 mM dithiothreitol (Sigma-Aldrich, St. Louis, MO, USA) and 30 mM EDTA (Boston Bioproducts, Boston, MA, USA), respectively. The lamina propria was subsequently exposed and digested with 333 μg/ml Liberase TL (Roche, Indianapolis, IN, USA) in DMEM (Gibco Life Technology, Gaithersburg, MD, USA) containing 5% fetal bovine serum (Atlanta Biologicals, Flowery Branch, GA, USA) for 100 min at 37°C in a 5% CO_2_ humidified incubator. All cells digested from tissue were passed through a 70 µm nylon cell strainer (Fisher Scientific) and then centrifuged (density gradient centrifugation) with OptiPrep (ρ = 1.055 g/ml) to yield DCs or Percoll (3 ml of 44% Percoll overlaid upon 3 ml of 67% Percoll) to yield T cells. Purified DCs and T cells were then stained and analyzed by FACSCalibur flow cytometer (BD Bioscience) followed by FlowJo software (Tree Star).

### DC and T Cell Activation

Dendritic cells in lamina propria were freshly prepared and sorted by flow cytometry (CD11c^+^MHCII^+^ as gate for DCs). Murine STING agonists (c-di-GMP) (Invivogen, San Diego, CA, USA) in designated concentration were incubated with DCs (3.5 × 10^4^/well) in 96-well plates for 3 days. Lipofectamine 2000 (Life Technologies, Invitrogen, Carlsbad, CA, USA) was used for transfection of c-di-GMP. Same volumes of c-di-GMP and Lipofectamine 2000 (i.e., 1:1 volume ratio) were mixed and incubated *in vitro* for 5 min at room temperature. The complex was subsequently added into cell culture system for transfection according to the manufacturer’s instruction. The cell pellet was collected for gene expression measurement.

CD4^+^ T cells freshly prepared from SILP and sorted by FACSCalibur (BD Bioscience) (CD3^+^ as gate for T cells) were cultured (2.5 × 10^5^/well) and stimulated with plate-bound anti-CD3 antibody (10 μg/ml) and soluble anti-CD28 antibody (1 μg/ml) for 3 days. The supernatant and cell pellets were collected for protein and gene expression measurement, respectively.

### OT-II Naive CD4^+^ T Cells and DCs Coculture Assay

Naïve CD4^+^ T cells were freshly prepared from spleen of transgenic OT-II mice and sorted as CD4^+^CD44^−^CD62L^+^ cells. Mucosal dendritic cells were freshly prepared from SILP and gated as CD11c^+^MHCII^+^ cells.

To activate DCs, 200 μg/ml chicken ovalbumin (Sigma-Aldrich, St. Louis, MO, USA) was added into the culture medium *in vitro*. Agonists of STING (c-di-GMP) (50 μg/ml) (Invivogen, San Diego, CA, USA), anti-IL-6 (25 ng/ml), recombinant IL-6 (20 ng/ml), anti-IL-1β (50 ng/ml), and recombinant IL-1β (20 ng/ml) (R&D Systems, Minneapolis, MN, USA) were incubated with OT-II naïve CD4^+^ T cells (2.5 × 10^5^/well) and DCs (3.5 × 10^4^/well) in 96-well plates for 3 days. The supernatant was collected for protein production measurement.

### Flow Cytometry

Isolated cells were incubated in 10% serum and Fc receptor-blocking antibody (clone NOD-15; catalog number 625801; BioLegend) for 15 min at 4°C and then stained with fluorescent-conjugated antibodies. PE/cy7-conjugated CD11c (HL3; 558079; BD PharMingen), BV510-conjugated I-A/I-E (M5/114.15.2; 107635; BioLegend), APC/cy7-conjugated CD11b (M1/70; 101225; BioLegend), PE-conjugated CD103 (M290; 557495; BD PharMingen), and APC-conjugated B220 (RA3-6B2; 103212; BioLegend) were used for DC staining. APC-conjugated CD3 (145-2C11; 100311; BioLegend), Pacific Blue-conjugated CD4 (GK1.5; 100428; BioLegend), PE-conjugated CD62L (MEL-14; 12-0621-81; eBioscience), and FITC-conjugated CD44 (IM7; 553133; BD PharMingen) were used for T cell staining. Cells were analyzed on FACSCalibur flow cytometer (BD Bioscience) followed by FlowJo software (Tree Star).

### DCs Sorting Strategy

Cells from lamina propria, MLNs, or spleen were prepared according to the previous step. FSC/SSC gating was initially employed to exclude debris and identify cell population of interest, followed by DAPI^−^ to exclude dead cells and/or CD3^−^ to exclude T cells. For DCs from lamina propria, CD11c^int/hi^MHCII^+^ were subsequently used to yield all DCs, which were then separated into CD103^+^ or CD103^−^ subpopulations according to their CD103 expression. The co-expression of CD11b and CD103 on DCs were analyzed as well (Figure S1 in Supplementary Material). For DCs from MLNs or spleen, CD11c^+^CD103^+^ was subsequently used to identify CD103^+^ DCs in respective organs (Figure S2 in Supplementary Material).

### Confocal Imaging

To visualize the vascular system, 100 μg Alexa Flour 647-conjugated wheat germ agglutinin (WGA) (Molecular Probes, Invitrogen, Carlsbad, CA, USA) was injected (i.v.) 7 min before imaging. Mice were sacrificed and tissues were immediately removed, opened by longitudinal incision, and rinsed with PBS. Living tissues were imaged with an A1R-A1 confocal microscope (Nikon, Melville, NY, USA), and 3D reconstructions were accomplished with Volocity software (PerkinElmer, Waltham, MA, USA).

### *Salmonella enterica* Serovar *Typhimurium* Infection

For *S. enterica* infection, food and water were withdrawn 4 h before the oral gavage with 200 μl PBS containing 1 × 10^9^ CFU of naturally streptomycin resistant *S. enterica* (SL1344). Water was immediately resumed, and food was provided 2 h post inoculation. Mice were sacrificed 24 h post infection, and the small intestine was removed for cell sorting. Liver, spleen, and feces were collected for bacterial load calculation. To measure bacterial load, the liver and spleen were cut into pieces, and homogenized in 5 ml PBS. Feces were homogenized in 5 ml PBS as well. After serial dilution, the homogenate was spread onto streptomycin-containing LB plate that was then incubated at 37°C overnight. CFU was counted and calculated in the next morning. All *Salmonella*-related experiment was conducted within the Bio-Safety Level 2 facility of Nanjing University in China.

### Gene Expression and Protein Production Measurement

Qiagen RNeasy kit was adopted for the extraction of RNA from all cell types and tissues. Subsequently, iScript cDNA synthesis kit (Bio-Rad) was used for synthesis of cDNA, and iQSYBR Green Supermix kit (Bio-Rad) was used for real-time PCR in Bio-Rad CFX96 Real-Time PCR Detection System according to the manufacturer’s instruction. *Gapdh* served as the house-keeping gene. The endpoint used in the real-time PCR quantification, *C*_t_, is defined as the PCR cycle number that crosses an arbitrarily placed signal threshold. Gene expression was calculated using $2^{-\Delta C_{\text{t}}}$ method, i.e., each well elicited a value of expression ratio by calculating $2^{-\left(C_{\text{t}}\left(target\right)-C_{\text{t}}\left(Gapdh\right)\right)}$, and each value was presented in bar graph.

Primers for murine samples were as follows: *Il6* forward, 5′-tagtccttcctaccccaatttcc-3′, and reverse, 5′-ttggtccttagccactccttc-3′; *Il10* forward, 5′-gctcttactgactggcatgag-3′, and reverse, 5′-cgcagctctaggagcatgtg-3′; *Il17a* forward, 5′-tttaactcccttggcgcaaaa-3′, and reverse, 5′-ctttccctccgcattgacac-3′; *Tnf* forward, 5′-caggcggtgcctatgtctc-3′, and reverse, 5′-cgatcaccccgaagttcagtag-3′; *Ifnb1* forward, 5′-ggcagatgtcctcaactgctc-3′, and reverse, 5′-gaccaccatccaggcgtag-3′; *Ifng* forward, 5′-acagcaaggcgaaaaaggatg-3′, and reverse, 5′-tggtggaccactcggatga-3′; *Il1b* forward, 5′-cacctctcaagcagagcacag-3′, and reverse, 5′-gggttccatggtgaagtcaac-3′; *Il4* forward, 5′-ggcattttgaacgaggtcaca-3′, and reverse, 5′-gacgtttggcacatccatctc-3′; *Il23a* forward, 5′-ccaatgtttccctgactttcca-3′, and reverse, 5′-aagtgtggtagcgaggaagca-3′; *Tgfb1* forward, 5′-gctaatggtggaccgcaacaac-3′, and reverse, 5′-cactgcttcccgaatgtctgac-3′; and *Gapdh* forward, 5′-aggtcggtgtgaacggatttg-3′, and reverse, 5′-ggggtcgttgatggcaaca-3′. Primers for human samples were as follows: *IL6* forward, 5′-ccttcggtccagttgccttct-3′, and reverse, 5′-ccagtgcctctttgctgctttc-3′; *IL17A* forward, 5′-cgaaatccaggatgccc-3′, and reverse, 5′-gacaccagtatcttctccag-3′; *TNF* forward, 5′-gcccctcccagttctagttc-3′, and reverse, 5′-aaagttggggacacacaagc-3′; and *GAPDH* forward, 5′-ggtgaaggtcggagtcaacg-3′, and reverse, 5′-caaagttgtcatggatgacc-3′.

Concentration of IL-10, IL-6, IL-17A, IFN-γ, and IL-4 in cell culture supernatant was detected with commercial enzyme-linked immunosorbent assay kit (eBioscience, San Diego, CA, USA).

### Statistic Analysis

All statistical tests were performed with GraphPad Prism Software (version 5.01; GraphPad, San Diego, CA, USA). All analyses were two-tailed, and differences were considered statistically significant when *p*-value < 0.05. Bars indicate mean ± SD. Student’s *t*-test was used for comparisons between two groups, while Kruskal–Wallis non-parametric test was used for comparisons between multiple groups. Correlation analysis was performed using linear regression model that yielded *R*^2^ values. Survival rate was compared using log-rank test. All experiments were repeated at least three times.

## Results

### Small Intestine Classical DCs Express CD103 and Elicit T Cell Responses

Dendritic cells are heterogeneous in origin. Distinct subpopulations of DCs are associated with specific functions in mucosal immunity. Recently, *Zbtb46* has been identified as a cDC-specific gene and their committed progenitor (17, 18). By using *Zbtb46*^GFP^ reporter mice, we revealed a remarkable co-expression pattern of Zbtb46 and CD103 in DCs in SILP (Figures 1A,B), suggesting that the small intestine cDCs predominantly expressed CD103. By contrast, the majority of CD11c^int^CD103^−^ cells expressed B220 but not CD11b (Figure 1B), suggesting they were predominantly plasmacytoid DCs (pDCs).

**Figure 1:** Mucosal classical dendritic cells (cDCs) express CD103 and elicit Th17 responses. **(A)** Co-expression of CD103 and Zbtb46 on CD11c^+^MHCII^+^ DCs in SILP. **(B)** Zbtb46, B220, and CD11b expression on CD11c^hi^CD103^+^ (G1) and CD11c^int^CD103^−^ cells (G2) in SILP. Representative of three independent experiments (*n* = 5). **(C)** IL-17A production during antigen-specific T cell activation by cDCs. CD11c^+^MHCII^+^CD103^+^ cDCs were isolated from either small intestinal lamina propria, spleen, or MLN, and were cocultured with splenic CD4^+^CD62L^+^CD44^−^ naïve T cells from OT-II transgenic mice in the presence of OVA for 3 days *in vitro*. Representative of three independent experiments (*n* = 4). **(D)** IL-17A, IL-10, IFN-γ, and IL-4 production during antigen-specific T cell activation by cDCs upon the activation of stimulator of interferon genes (STING) agonist. cDCs were isolated from SILP and were transfected using Lipofectamine with c-di-GMP followed by coculture with splenic CD4^+^CD62L^+^CD44^−^ naïve T cells from OT-II transgenic mice in the presence of OVA for 3 days *in vitro*. Representative of three independent experiments (*n* = 5). **(E)** IL-17A production during antigen-specific T cell activation by cDCs or pDCs upon the activation of STING agonist. Cells were prepared as described in panel **(D)**. Representative of three independent experiments (*n* = 5). **(F)** IL-17A and IL-10 production during antigen-specific T cell activation by CD103^+^ cDCs. Cells were prepared as described in panel **(D)** and were incubated with anti-IL-6, recombinant IL-6, anti-IL-1β, and recombinant IL-1 β in the presence of OVA for 3 days *in vitro*. Representative of three independent experiments (*n* = 5). **(G)** STING production in spleen and colon tissue of WT and *Tmem173^−/−^* (^−/−^) mice. **(H)** Fold change of *Il6, Ifnb1, Tnf, Il1b, Il10, Il23a*, and *Tgfb1* gene expression in cDCs of *Tmem173^−/−^* mice in response to STING activation. C57BL/6 and *Tmem173^−/−^* mice were injected (i.p.) with PBS or c-di-GMP at days −1, −3, and −5, and cDCs were then isolated from SILP (*n* = 4). **(I)** IL-17A, IL-10, IFN-γ, and IL-4 production during antigen-specific T cell activation by cDCs upon the stimulation of STING. cDCs were isolated from SILP of C57BL/6 or *Tmem173^−/−^* mice and transfected with c-di-GMP followed by coculture with splenic CD4^+^CD62L^+^CD44^−^ naïve T cells from OT-II transgenic mice in the presence of OVA for 3 days *in vitro* (*n* = 4). Abbreviations: SILP, small intestine lamina propria; MLN, mesenteric lymph node; ND, not detectable; pDC, plasmacytoid DC.

To compare the capacity of antigen presentation between cDCs from spleen, MLN and SILP, we established an *in vitro* coculture system consist of cDCs (defined as CD11c^+^MHCII^+^CD103^+^) and OT-II TCR transgenic CD4^+^CD62L^+^CD44^−^ naïve T cells. cDCs from SILP elicited significantly stronger immune responses (represented by IL-17A secretion) compared with CD103^+^ DCs from spleen and MLN upon OVA stimulation (Figure 1C; Figures S1 and S2 in Supplementary Material).

To determine whether mucosal cDCs responded to STING-mediated signaling, we transfected the microbial second messenger c-di-GMP into cDCs and cocultured with OT-II naïve T cells in the presence of OVA. We found that mucosal immunity required cDCs-mediated antigen presentation, since T cells failed to secrete either IL-17A or IL-10 in the absence of cDCs. Furthermore, we found that c-di-GMP-initiated STING signaling induced Th1 (IFN-γ)/Th2 (IL-4)/Th17 (IL-17A) immune responses (19–21) while inhibited IL-10 production *via* OVA-activated cDCs (Figure 1D).

To compare the capacity of inducing Th17 immunity by cDCs or pDCs (defined as CD11c^int^MHCII^+^CD103^−^B220^+^, Figure S1 in Supplementary Material) during STING activation, we transfected c-di-GMP into cDCs or pDCs isolated from SILP and cocultured with OT-II naïve T cells in the presence of OVA. We found that cDCs elicited significantly more IL-17A secretion compared with pDCs. Moreover, c-di-GMP transfection into pDCs failed to mount Th17 immunity in gut (Figure 1E), suggesting cDCs in SILP were the major STING signaling cells involved in Th17 differentiation.

To determine the mechanism of STING-mediated mucosal immunity, we added anti-IL-6 and recombinant IL-6 into the coculture system. Blocking of IL-6 reversed IL-17A induction and rescued IL-10 reduction by c-di-GMP, while recombinant IL-6 was able to synergize with c-di-GMP in inducing Th17 responses (Figure 1F). Similarly, blocking of IL-1β or recombinant IL-1β inhibited or rescued IL-17A production by c-di-GMP (Figure 1F). Together, we identified that STING signaling contributed to Th17 generation through the induction of IL-6/IL-1β secretion by mucosal cDCs.

We next sought to determine the obligatory role of STING in response to cyclic dinucleotides in gut. We generated *Tmem173 (Sting)*-deficient mice using CRISPR-Cas9 technology (Figure 1G). *Tmem173*-deficient mucosal cDCs expressed less *Il6, Ifnb1, Il1b*, and *Il23a* but more *Il10* mRNA in steady state, and more importantly, failed to express higher inflammatory *Il6, Ifnb1, Tnf, Il1b, Il23*, and *Tgfb1* mRNA levels or lower *Il10* mRNA level after being stimulated with c-di-GMP *in vivo* (Figure 1H). By contrast, *Tmem173*-deficient mucosal pDCs expressed similar mRNA levels of all above cytokines to C57BL/6 and were unresponsive to c-di-GMP stimulation except for the *Tnf* and *Tgfb1* mRNA expression (Figure S3 in Supplementary Material).

Furthermore, we isolated and stimulated cDCs from SILP of C57BL/6 control and *Tmem173*-deficient mice with c-di-GMP and cultured them with OT-II naïve T cells in the presence of OVA. We found that *Tmem173*-deficient cDCs induced significantly less IL-17A in steady state and were unable to induce IL-17A production during antigen-specific T cell activation compared with C57BL/6 control cDCs. By contrast, *Tmem173*-deficient mucosal cDCs induced significantly more IL-10 secretion during antigen-specific T cell activation. We observed that promotion of Th1 and Th2 responses by c-di-GMP is independent of STING signaling (Figure 1I), although other vaccine adjuvants (e.g., chitosan) required STING to elicit Th1 immunity (22), and Th1 suppression of STING-mediated DNA sensing was reported as well (23). Together, these experiments demonstrated that mucosal Th17 polarization by cDCs was entirely dependent on STING signaling.

### STING Triggers Th17 Differentiation in Gut

To further demonstrate the effect of STING signaling on mucosal immunity, we performed repeated injection of foreign cyclic dinucleotides into mice. The *ex vivo* analysis of lamina propria cDCs showed that c-di-GMP induced a significant elevation in *Il6, Il1b, Ifnb, Tnf, Il23a*, and *Tgfb1* mRNA expression and a significant decline in *Il10* mRNA expression (Figure 2A). By contrast, c-di-GMP failed to regulate cytokine mRNA expression in pDCs except *Tnf* and *Tgfb1* that were increased by c-di-GMP (Figure S4 in Supplementary Material). We further observed the generation of IL-17A-expressing T cells using *Il17a*^GFP/GFP^ reporter mice with repeated c-di-GMP *in vivo* stimulation. Both confocal imaging and flow cytometry revealed a significant increase in Th17 cells in small intestine, Peyer’s patch, MLN, spleen except colon (Figure 2B). Notably, a relatively higher proportion of Th17 cells was identified in SILP and Peyer’s patch compared with other sites (Figure 2B), suggesting that mucosa was the predominant arena of Th17 differentiation triggered by STING signaling.

**Figure 2:** Stimulator of interferon genes (STING) triggers Th17 differentiation in gut. **(A)** Fold change of *Ifnb1, Il6, Il1b, Tnf, Il10, Il23a*, and *Tgfb1* gene expression in classical dendritic cells from small intestinal lamina propria in response to STING agonist. PBS or c-di-GMP was injected (i.p.) before sacrifice (*n* = 5). **(B)** Confocal imaging (left) and flow cytometry analysis (middle) of IL-17A production together with IL-17A-expressing cells (right) in small intestine lamina propria, Peyer’s patch, colon, mesenteric lymph node and spleen in response to the activation of STING signaling. *Il17a*^GFP/GFP^ reporter mice were injected (i.p.) with c-di-GMP on day −5, day −3, and day −1, followed by wheat germ agglutinin (WGA) injected (i.v.) 7 min before sacrifice. Fold change was calculated according to flow cytometry analysis. Representative of three independent experiments (*n* = 3). Scale bars, 50 µm.

### CD103^+^ cDCs Are Essential for Mucosal Immunity to Cyclic Dinucleotides

To determine the essential role of cDCs in shaping mucosal immunity, we established *Zbtb46* bone marrow chimeric mice in which hematopoietic system was derived from *Zbtb46*^GFP^ mice. Both epithelium and hematopoietic cells expressed GFP signaling in *Zbtb46*^GFP^ mice (Figure 3A left), whereas Zbtb46-expressing cDCs in small intestine were clearly identified after bone marrow transplantation in recipient C57BL/6 mice by confocal imaging (Figure 3A right). Similarly, *Zbtb46*^DTR^ bone marrow chimeric mice were developed, in which recipient C57BL/6 mice received whole body irradiation followed by bone marrow cells from *Zbtb46*^DTR^ mice. Two DT injections significantly depleted cDCs population in lamina propria while not affecting CD103^−^CD11b^+^CD11c^+^MHCII^+^ myeloid phagocytes. Interestingly, foreign cyclic dinucleotides induced CD103^+^CD11c^+^MHCII^+^ subset predominantly expressing CD11b^+^ (Figure 3B upper panel) even in cDCs-depleted mice (Figure 3B lower panel), implying c-di-GMP might stimulate *de novo* DC differentiation from precursors.

**Figure 3:** Mucosal cDCs are essential for immune responses to cyclic dinucleotides. **(A)** Confocal imaging of Zbtb46^+^ cells in small intestine lamina propria (SILP). GFP expression in *Zbtb46*^GFP^ mice (left) or in recipient C57BL/6 mice that received bone marrow cells from *Zbtb46*^GFP^ mice after whole body irradiation (right). Recipient WGA was injected (i.v.) 7 min before sacrifice. Representative of three independent experiments (*n* = 3). **(B)** Depletion of mucosal cDCs from *Zbtb46*^DTR^ bone marrow chimeric mice. Recipient C57BL/6 mice received bone marrow cells from *Zbtb46*^DTR^ mice after whole body irradiation. DT was injected (i.p.) on day −3 and day −1, and c-di-GMP was injected (i.v.) 18 h before analysis. Representative of three independent experiments (*n* = 3). **(C)** Fold change of *Il17a, Ifng, Il10*, and *Il4* gene expression in CD4^+^ T cells in *Zbtb46*^DTR^ bone marrow chimeric mice. Mice were prepared as described in panel **(B)**. CD3^+^CD4^+^ T cells were isolated from SILP and were stimulated *in vitro* by anti-CD3 and anti-CD28 for 3 days (*n* = 5). Abbreviations: DT, diphtheria toxin; WGA, wheat germ agglutinin; cDC, classical dendritic cell.

In the presence of cDCs, lamina propria CD4^+^ T cells expressed higher *Il17a, Ifng*, and *Il4* mRNA and lower *Il10* mRNA levels upon c-di-GMP stimulation. By contrast, after depletion of cDCs by DT injections, lamina propria CD4^+^ T cells were unable to express *Il17a, Ifng, Il4*, or *Il10* mRNA, suggesting that cDCs are essential for mediating T cell immunity in gut (Figure 3C).

### STING Correlates With Intestinal Inflammation and Controls T Cell Polarization

Inappropriate sensing of self or foreign DNA has been associated with imbalanced host immune responses. STING-controlled signaling events are involved in human autoimmune diseases. To determine the correlation between STING expression in lamina propria and intestinal inflammation, we recruited human samples from Crohn’s patients and compared them to samples from patients receiving ileostomy closure. The density of immunohistochemistry staining of STING was highest in Crohn’s lesion, moderate in Crohn’s para-lesion, and lowest in control (Figure 4A). Linear regression analysis demonstrated a positive correlation between the severity of inflammation and optical density of STING expression (Figure 4A). STING-controlled IRF3 activation was also found in Crohn’s lesion compared with para-lesion and control (Figure 4B). Simultaneously, we revealed a significant correlation of *IL17A, TNF*, and *IL6* mRNA expression in tissue to STING density (Figure 4C). Furthermore, we demonstrated that clinical CDAI score was in parallel to STING expression in gut as well (Figure 4D). Together, these data suggested the pro-inflammatory involvement of STING signaling in human Crohn’s disease.

**Figure 4:** Stimulator of interferon genes (STING) recognizes cyclic dinucleotides and correlates with intestinal inflammation. **(A)** Correlation between severity of intestinal inflammation (HE staining) and expression level of STING (IHC staining) (left) in human gut was analyzed (right). Human intestine specimens were collected at normal site from non-Crohn’s patients (control) and at para-lesions as well as lesions from Crohn’s patients. The optical density of STING was measured by Image J in IHC staining slides. Each symbol represents an individual patient. **(B)** Activation of STING signaling in gut of Crohn’s patients. Human intestine specimens were collected as described in panel **(A)**. **(C,D)** Correlation of cytokine expression in tissue samples **(C)** and clinical CDAI score **(D)** to the expression level of STING. The optical density of STING was measured by Image J in IHC staining slides. Each symbol represents an individual patient. Pathological slides, 100× amplification. Abbreviations: HE, hematoxylin and eosin; IHC, immunohistochemistry; CD, Crohn’s disease; CDAI, Crohn’s disease activity index.

### STING-Regulated Th17 Responses Help Host Defense Against *Salmonella* Infection

*Salmonella enterica* serovar *Typhimurium* induces Th1 and Th17 responses that result in mucosal inflammation and diarrhea (24, 25). We utilized *Salmonella* infection model to elucidate the role of STING-controlled Th17 responses in antimicrobial infections. *Tmem173*-deficient mice exhibited significantly decreased survival rate compared with C57BL/6 mice after *Salmonella* infection (*p* = 0.01) (Figure 5A). By oral gavage with *Salmonella* in *Il17a*^GFP/GFP^ reporter mice, CD4^+^IL-17A^+^ T cells increased in lamina propria (Figure 5B). By analyzing DC subpopulations in lamina propria, we found that cDCs (CD11c^+^CD103^+^) were recruited by *Salmonella* in C57BL/6 mice. By contrast, cDCs remained similar in lamina propria of *Tmem173*-deficient mice to those found in uninfected littermates (Figure 5B).

**Figure 5:** Stimulator of interferon genes controls Th17 responses for host defense against *Salmonella* infection. **(A)** Survival curves of C57BL/6 and *Tmem173^−/−^* mice infected with *Salmonella*. Mice were inoculated orally with *Salmonella* and observed for 7 days after infection (*n* = 8). Statistical significance (*p* = 0.01) was determined by log-rank test. **(B)** Flow cytometry analysis of cDCs (top) and IL-17A-expressing CD4^+^ T cells (bottom) in small intestine lamina propria (SILP) during *Salmonella* infection. C57BL/6, *Tmem173^−/−^*, and *Il17a*^GFP/GFP^ reporter mice were inoculated orally with *Salmonella* 24 h before sacrifice. Representative of three independent experiments (*n* = 4). **(C)** IL-17A production during antigen-specific T cell activation by cDCs or pDCs isolated from either uninfected (Contl.) or *Salmonella-*infected (Sal.) C57BL/6 mice. DCs were isolated from SILP and were cocultured with splenic CD4^+^CD62L^+^CD44^−^ naïve T cells from OT-II transgenic mice in the presence of OVA for 3 days *in vitro*. Representative of three independent experiments (*n* = 4). **(D)** Fold change of *Il6, Il1b, Tnf, Ifnb1, Il10, Il23a*, and *Tgfb1* gene expression in cDCs as well as IL-17A, IFN-γ, and IL-4 production by CD4^+^ T cells after *Salmonella* infection. C57BL/6 and *Tmem173^−/−^* mice were infected with *Salmonella* as described in panel **(B)**. cDCs and CD4^+^ T cells were isolated from SILP. CD4^+^ T cells were then stimulated *in vitro* by anti-CD3 and anti-CD28 for 3 days (*n* = 5). **(E)** Bacterial load in liver after *Salmonella* infection (*n* = 3). C57BL/6 and *Tmem173^−/−^* mice were infected with *Salmonella* as described in panel **(B)**. Abbreviations: ND, not detectable; pDC, plasmacytoid DC; cDC, classical dendritic cell.

To compare the Th17 immunity induced by different DC subpopulations during *Salmonella* infection, cDCs (CD11c^+^MHCII^+^CD103^+^B220^−^) or pDCs (CD11c^int^MHCII^+^CD103^−^B220^+^CD11b^−^) isolated from SILP of uninfected or *Salmonella*-infected C57BL/6 mice were cocultured with OT-II naïve T cells *in vitro* in the presence of OVA (Figure S5 in Supplementary Material). *Salmonella*-infected cDCs elicited significantly more IL-17A production compared with *Salmonella*-infected pDCs or uninfected cDCs (Figure 5C). These data indicated that cDCs in SILP were the major STING signaling cells involved in mucosal Th17 differentiation during *Salmonella* infection.

In support of a direct regulation of mucosal DCs function by *Salmonella*, we found that cDCs in C57BL/6 mice expressed significantly more *Il6, Il1b, Tnf, Ifnb1, Il23a*, and *Tgfb1* mRNA and less *Il10* mRNA after *Salmonella* infection. However, *Tmem173*-deficient cDCs demonstrated naturally decreased level of *Il6* and *Ifnb1* mRNA and increased level of *Il10* mRNA. More importantly, *Tmem173*-deficient cDCs were unable to respond to *Salmonella* except elevated *Tgfb1* expression (Figure 5D). By contrast, lamina propria pDCs of C57BL/6 and *Tmem173^−/−^* mice demonstrated similar cytokine profiles at steady state and were unresponsive to *Salmonella* infection except elevated *Tgfb1* mRNA expression (Figure S6 in Supplementary Material).

Consistently, *Tmem173*-deficient CD4^+^ T cells produced naturally less IL-17A and failed to respond with the induction of Th17 cells to infection (Figure 5D). By contrast, *Salmonella* induced IFN-γ production by CD4^+^ T cells independent of STING. More importantly, we observed that *Tmem173*-deficient mice were unable to defend against *Salmonella* infection in consequence as indicated by the significantly increased bacterial load in liver, spleen, and feces compared with C57BL/6 mice (Figure 5E). Together, these data indicated that STING signaling was required as an integral mechanism of mucosal immune defenses to foreign pathogens.

## Discussion

Our study revealed that STING signaling activates IL-17A while inhibits IL-10 production by adaptive T cells during antigen presentation in gut. Mucosal CD103^+^ cDCs that express the transcription factor *Zbtb46* are required for Th17 development in response to bacterial second messenger in small intestine. In addition, STING-IRF3 signaling correlates with disease activity and mucosal inflammation severity in patients with Crohn’s disease. Since Th17 axis has been implicated as a hallmark of infectious diseases and inflammatory bowel diseases (IBD), our discovery of STING-controlled Th17 immunity provides new insights into the pathogenesis of IBD and potential interventional target for future therapy.

Dendritic cells are responsible for T cell polarization. The ability of inducing T cell differentiation varies between subgroups of DCs. CD103^+^ DCs are previously found to mainly induce Tregs and suppress Th17 responses to gut bacteria (26), although inconsistent findings report that CD103^+^ DCs are capable but dispensable to induce Th17 cells in response to certain commensals (27, 28) We discovered that CD103^+^ cDCs are indispensable and capable to induce both IL-10 and IL-17A expression upon antigen stimulation, in which STING determines a Th17-dominated outcome of antigen presentation by cDCs in gut although specific mechanism remains unclear. Recent studies have reported that STING activation in T cells triggers apoptosis (29–31), suggesting diverse functions of STING that controls inflammatory events in innate immunity while inhibits lymphocytes proliferation in adaptive immunity. Interestingly, the induction of Th17 populations by cyclic dinucleotides was phenomenal in mucosa-associated immune system, implying that intestinal cDCs utilize STING for mucosal protection.

Th17 differentiation requires a series of cytokines including IL-6, TGF-β, IL-1β, and IL-23. Among them, IL-6 has been well recognized as the critical elements to induce Th17 differentiation (32–34). In addition, IL-1 signaling was reported to be critical for Th17 polarization in mice (35). Nevertheless, the role of IL-1β in Th17 induction seems controversial in human. IL-1β can induce Th17 maturation and simultaneously give rise to Th17/Th1 complex and Th1 cells (36). IL-1β is required for two types of pathogen-induced human Th17 cells with distinct effector functions (37). In our study, we demonstrated that both IL-6 and IL-1β are central regulators of STING-mediated mucosal Th17 immunity.

To elucidate the consequence of STING activation in mucosal cDCs, we identified STING as a target for immune evasion of enteroinvasive pathogens. We demonstrated that *Salmonella* recruits cDCs and induces significant Th17 responses in mucosal immune system that are entirely dependent on STING signaling. Furthermore, the absence of STING is associated with *Salmonella* escape from gut to liver, suggesting that STING is essential for host to prevent bacteria translocation, which is consistent to previous findings in lung (38). Nevertheless, the underlying mechanism by which pathogens regulate STING remains elusive. We hypothesize that other pathogen recognition receptor-mediated signaling could interact with STING to compete for mucosal immunity.

In conclusion, our study discovers that microbial cyclic dinucleotides recognition can drive mucosal Th17 generation. The identification of STING as a decisive element of T cell differentiation may explain why mucosal DCs are able to trigger both immune defenses through Th17 cells and immune regulation by IL-10 to shape individual reaction to gut microbiota. Polymorphisms in signaling pathways that involve Th17 polarization and IL-10 contribute to the risk profiles of IBD and other autoimmune diseases (39). Therefore, the identification of STING-induced Th17 responses and STING-suppressed IL-10 production would help to elucidate the causal relationship between generic variants and nucleic acid recognition by mucosal DCs for host defenses in gut.

## Data Availability Statement

The raw data supporting the conclusions of this manuscript will be made available by the authors, without undue reservation, to any qualified researcher.

## Ethics Statement

This study was carried out in accordance with the recommendations of Guidelines for Clinical Trials by the Ethics Committee of Nanjing Drum Tower Hospital. The protocol was approved by the Ethics Committee of Nanjing Drum Tower Hospital. All subjects gave written informed consent in accordance with the Declaration of Helsinki. This study was carried out in accordance with the recommendations of Guidelines for Animal Experiment by the Ethics Committee of Nanjing Drum Tower Hospital. The protocol was approved by the Ethics Committee of Nanjing Drum Tower Hospital.

## Author Contributions

Conceptualization: WG. Methodology: SL, QX, and QR. Investigation: SL, QX, XW, FS, QH, JW, and MW. Writing—original draft: SL and QX. Writing—review and editing: WG; funding acquisition: SL and WG. Resources and supervision: QR and WG.

## Conflict of Interest Statement

The authors declare that the research was conducted in the absence of any commercial or financial relationships that could be construed as a potential conflict of interest.

## Supplementary Material

Figure S1 Lamina propria DCs separation strategy by flow cytometry. Cells from small intestine lamina propria were prepared according to the description in Section “Materials and Methods” and were sorted using FACSCalibur flow cytometer (BD Bioscience) and analyzed by FlowJo software (Tree Star). Initially, FSC/SSC gating was employed to exclude debris and identify cell population of interest, followed by DAPI^−^ to exclude dead cells and CD3^−^ to exclude T cells. Subsequently, CD11c^int/hi^MHCII^+^ was used to yield all DC populations, which were then separated into CD103^+^ or CD103^−^ population according to their CD103 expression. The expression of B220 in CD103^+^ and CD103^−^ populations were analyzed. The co-expression of CD11b and CD103 on DCs was analyzed as well.

Figure S2 Separation strategy of DCs in mesenteric lymph nodes and spleen by flow cytometry. Cells from mesenteric lymph nodes or spleen were prepared according to the description in Section “Materials and Methods” and were sorted using FACSCalibur flow cytometer (BD Bioscience) and analyzed by FlowJo software (Tree Star). Initially, FSC/SSC gating was employed to exclude debris and identify cell population of interest, followed by DAPI^−^ to exclude dead cells. CD11c^+^CD103^+^ was subsequently used to identify CD103^+^ DCs in respective organs.

Figure S3 Cytokine expression of *Tmem173*-deficient pDCs in response to cyclic dinucleotides. Fold change of *Il6, Ifnb1, Tnf, Il1b, Il10, Il23a*, and *Tgfb1* gene expression in plasmacytoid DCs (pDCs) of *Tmem173^−/−^* mice in response to cyclic dinucleotides. C57BL/6 and *Tmem173^−/−^* mice were injected (i.p.) with PBS or c-di-GMP at day −1, −3, and −5, and pDCs were then isolated from small intestine lamina propria (*n* = 4).

Figure S4 *Ex vivo* analysis of cytokine expression by plasmacytoid DCs (pDCs) in response to cyclic dinucleotides. Fold change of *Ifnb1, Il6, Il1b, Tnf, Il10, Il23a*, and *Tgfb1* gene expression in pDCs from small intestinal lamina propria in response to cyclic dinucleotides. PBS or c-di-GMP was injected (i.p.) before sacrifice (*n* = 5).

Figure S5 Lamina propria DCs separation strategy during *Salmonella* infection by flow cytometry. Cells from small intestine lamina propria were prepared according to the description in Section “Materials and Methods” and were sorted using FACSCalibur flow cytometer (BD Bioscience) and analyzed by FlowJo software (Tree Star). Initially, FSC/SSC gating was employed to exclude debris and identify cell population of interest, followed by DAPI^−^ to exclude dead cells. Subsequently, CD11c^int/hi^MHCII^+^ was used to yield all DC populations, which were then separated into CD103^+^ or CD103^−^ population according to their CD103 expression. The expression of B220 and CD11b in CD103^+^ and CD103^−^ populations were further analyzed.

Figure S6 Cytokine expression of *Tmem173*-deficient plasmacytoid DCs (pDCs) in response to *Salmonella* infection. Fold change of *Il6, Ifnb1, Tnf, Il1b, Il10, Il23a*, and *Tgfb1* gene expression in pDCs of *Tmem173^−/−^* mice in response to *Salmonella* infection. C57BL/6 and *Tmem173^−/−^* mice were mice inoculated orally with *Salmonella* 24 h before sacrifice, and pDCs were then isolated from small intestine lamina propria (*n* = 4).
